This article has been retracted.

# Analysis of psychological characteristics and emotional expression based on deep learning in higher vocational music education

**DOI:** 10.3389/fpsyg.2022.981738

**Published:** 2022-09-23

**Authors:** Xin Liu

**Affiliations:** Henan Vocational College of Arts, Zhengzhou, Henan, China

**Keywords:** sentiment analysis, higher vocational music education, deep learning, review text, psychological characteristics and emotional

## Abstract

Sentiment analysis is one of the important tasks of online opinion analysis and an important means to guide the direction of online opinion and maintain social stability. Due to the multiple characteristics of linguistic expressions, ambiguity, multiple meanings of words, and the increasing speed of new words, it is a great challenge for the task of text sentiment analysis. Commonly used machine learning methods suffer from inadequate text feature extraction, and the emergence of deep learning has brought a turnaround for this purpose. In this paper, we investigate the problem of text sentiment analysis using methods related to deep learning. In order to incorporate user and product information in a more diverse way in the model, this paper proposes a model based on a deep bidirectional long-and short-term memory network-self-attention mechanism-custom classifier. The model first identifies contextual associations and acquires deep text features through a deep bidirectional long- and short-term memory network and then captures important features in the text using a self-attentive mechanism. The model finally combines user information and product information to build a custom classifier module and uses context-aware attention mechanisms to assign specific parameters to user information and product information, which improves the performance of the model on public datasets compared with current common models. The results show that the accuracy of the algorithm in this paper is high, and it is about 5% lower than the traditional algorithm. The method can reduce the number of iterations and the running time of the algorithm.

## Introduction

At present, with the intensification of market competition, the increase of social information, the acceleration of life rhythm, and the increase of psychological crisis, traditional concepts, historical details, ethics, value orientation, etc. have all encountered unprecedented impacts, and adults will still be psychologically lost (Jung, 2015). What’s more, teenagers are at the stage of physiological and psychological development, and their physical and mental influences are even greater. As a special group, students in higher vocational colleges are exposed to social changes, inevitably facing severe challenges of adaptation and development, and their psychology is increasingly impacted and influenced. When these impacts and influences exceed students’ psychological endurance, they will bring many unstable factors to the school, which will lead students to neglect their studies and make it difficult for them to become talents. The analysis of higher vocational students’ psychological problems and the study of educational countermeasures are beneficial to the development of our mental health education for higher vocational students, and at the same time, it is of great significance to the goal of cultivating all-round qualified higher vocational students who meet the requirements of the new era (Liang, 2020).

As the top priority of higher vocational students’ analysis, text sentiment analysis has attracted a lot of attention in the field of natural language processing. The explosive growth of text data on the Internet and new linguistic features have brought great challenges to the task of text classification (Department of Human, 2016). At present, artificial intelligence technology represented by deep learning has performed well in solving text classification problems, so this paper uses deep learning related technologies in text sentiment analysis, hoping to obtain better classification performance, so as to better achieve As an important development direction in the field of artificial intelligence, deep learning of network public opinion supervision has achieved good results in computer vision, speech, text and other fields. The key is to analyze the overall sentiment bias of a comment text by extracting text features. This classification method is simple and direct. The most common analysis method for sentiment analysis of user comments is to perform document-level sentiment analysis on the text (Redeker et al., 2018).

Nowadays, although some scholars have used neural networks to extract text features and achieved good results, how to improve sentiment analysis for user reviews by mining deeper features of text and semantic association features has been a hot issue in research. Meanwhile, although many scholars have built sentiment analysis models based on deep learning methods and got good results for different scenarios, document-level sentiment analysis tasks for product reviews need to consider user data and product data on the basis of general sentiment analysis models in order to improve the analysis results (Li, 2021). This chapter introduces the research background of psychological feature analysis and sentiment expression in higher education music education and the practical significance of text sentiment analysis in recent years, and provides a detailed overview of the current status of research on psychological feature analysis and sentiment expression in higher education music education and the current status of text classification research, and outlines the main contents and organization of this thesis. Its innovations are (Tang, 2017).

This paper summarizes the research status of online public opinion and text sentiment classification methods based on deep learning, probes into the advantages and disadvantages of various classification methods, and introduces the text preprocessing process and related technologies used, several vector representation methods of texts and some basic models of common neural networks.

The experimental verification of various text sentiment classification models proves the superiority of the model proposed in this paper.

This paper studies the analysis of psychological characteristics and emotional expression based on deep learning in higher vocational music education. The structure is as follows.

The first chapter is the introduction. This part mainly expounds the research background and significance of psychological characteristics analysis and emotional expression based on deep learning in higher vocational music education, and puts forward the research purpose, method and innovation of this paper. The second chapter is a summary of relevant literature, summarizing its advantages and disadvantages, and putting forward the research ideas of this paper. The third chapter is the method part, focusing on the analysis of psychological characteristics and emotional expression in the combination of deep learning and higher vocational music education. The fourth chapter is the experimental analysis. In this part, experiments are carried out on data sets to analyze the performance of the model. Chapter five, conclusion and prospect. This part mainly reviews the main contents and results of this research, summarizes the research conclusions and points out the direction of further research.

## Related work

“Emotion” not only refers to a specific emotional state, but also refers to all the feelings related to the body, the mind, the senses, and the spirit, which are expressed through language. Therefore, Hochreiter proposed Long Short-Term Memory (LSTM), which determines how to use and update the information in the storage unit by capturing the long-term dependencies between sentences to obtain more permanent information (Hochreiter, 2021). It shows good performance in classification. Huang proposed a model for sentiment analysis of Chinese text using BiLSTM (Huang, 2018). Due to the use of multiple “gate” structures, it is more complex and has many parameters. Therefore, some scholars have improved LSTM and reduced its parameters. The proposed new model is called Gated Recurrent Neural Network (GRU). In order to better synthesize the context of the article, Cao uses the BiGRU model to classify Chinese texts. The model is simple, has few parameters, and has fast convergence speed, and also shows good performance in NLP (Cao, 2017). Since then, a large number of hybrid neural network classification models have appeared. Guo proposed to use a CNN-BiLSTM model for sentiment analysis, which has better accuracy compared to a single neural network approach (Guo, 2016). SobkowiczP proposed a public opinion system model based on social information network, and elaborated the four development stages of network public opinion and their correlations (Sobkowicz, 2017). Dang uses TF-IDF combined with word vector model to classify speech sentiment on the Internet (Dang, 2017). Xu applies opinion mining methods to cross-media analysis to detect and track emergencies, providing methodological support for the government and relevant administrative departments (Xu, 2021). The Hierarchical Attention Network model proposed by Yang for the sentence classification problem uses the attention mechanism to model sentences, which reduces the gradient disappearance problem generated by RNN when processing sequence data to a certain extent (Yang, 2020). The DeepMojo model proposed by Feibo has a good effect in the sentiment analysis task of text and emoji expressions (Feibo, 2019). Cho designs an adaptive memory and forget structure for each RNN unit, which can learn long-term and short-term features while reducing the risk of gradient dispersion (Cho, 2020).

Vigorous development of higher vocational education has become an important national policy in many countries. Under this circumstance, higher vocational colleges and universities are responsible for cultivating highly skilled talents which are urgently needed by the country, and qualified highly skilled talents need healthy psychological quality. In addition to cultivating students’ practical ability, higher vocational colleges must also make students have high moral character, rigorous and responsible spirit, good interpersonal communication and the ability to coordinate and cooperate in a group, the ability to adapt positively and the ability to solve problems, and the spirit of optimism toward life, lifelong learning and continuous innovation. The above-mentioned training contents are the needs of today’s social development. In this paper, we propose a design scheme for psychological profiling and emotional expression in higher education music education based on deep learning, and conduct a design scheme for deep learning and psychological profiling and emotional expression in higher education music education based on deep learning background. Information and effectively improve the accuracy of the sentiment multi-categorization task.

## Methodology

### CBOW model

The concept of distributed, the chief intention is to target the words in the high-dimensional space, and finally get the N-dimensional vector corresponding to the word through model training and finally the semantic relationship between words can be measured by calculating the distance between words. Word2Vec is a typical method of distributed representation of word vectors. The Word2Vec method has representation, CBOW. The specific model structure is shown in Figure 1.

**Figure 1:** Concrete model structure of CBOW model.

First, the first m words of the central word w and the one-hot representation of the next m words are projected into the hidden layer using the transfer matrix. In the hidden layer, unlike the traditional NNLM, the vectors are summed and averaged without activation to obtain the output of the hidden layer (Al-Shaher, 2020). The vectors in the hidden layer are fully concatenated and then fed to the output layer, which is activated using the Softmax function to obtain the final output. For training using the CBOW model, the optimization objectives to be maximized are shown in equation (1).


(1) $$J=\frac{1}{T}\underset{t=1}{\sum }\log p\left(w^{t}\right)|w^{\left(t-m\right)},\ldots w^{\left(t-1\right)},\ldots ,w^{\left(t+1\right)},\ldots ,w^{\left(t+m\right)}$$

### Skip-gram model

As can be seen from Figure 2, the Skip-gram model and the CBOW model work from opposite perspectives, such as the existing text sequence $\left(w_{t-n},\ldots ,w_{t-1},w_{t,}w_{t+1,}\ldots ,w_{t+n}\right)$, i represents the $w_{t}$th word in the sequence, $w_{t}$ represents the known word, the context within the defined window is $\left(w_{t-n},\ldots ,w_{t-1},w_{t,}w_{t+1,}\ldots ,w_{t+n}\right)$ and the window size isn. The model analyzes the known word $w_{t}$ and outputs the sequence with the highest probability as the context $\left(w_{t-n},\ldots ,w_{t-1},w_{t,}w_{t+1,}\ldots ,w_{t+n}\right)$. Although Word2Vec incorporates semantic information of words into the modeling process, Word2Vec only considers the semantic and logical connections of words within the window, but not the semantic and logical connections of words and words outside the window, which will undoubtedly cause inaccurate results. The Glove model mainly decomposes the co-occurrence matrix between words and words to achieve the global semantic overall linkage, and finally obtains a distributed representation of words (Kim and Choi, 2020). The degree of semantic similarity between words can be measured by calculating the distance between words.

**Figure 2:** Skip-gram model specific model structure.

Each element $X_{ij}$ of the co-occurrence matrix X in the Glove word vector model is the logarithm of the total number of co-occurrence of the words $w_{i}$ and $w_{j}$. The number of co-occurrence of the words $w_{i}$ and $w_{j}$ is calculated by the decay function $decay=\frac{1}{d}$. The total number of occurrences of word $w_{i}$ is calculated by$x_{i}=\underset{k}{\sum }x_{ik}$, and the probability of word $w_{j}$ occurring around $w_{i}$ is calculated by equation (2).


(2) $$p_{ij}=p\left(w_{j}|w_{i}\right)=\frac{x_{ij}}{x_{i}}$$

The approximate solution of $\log\left(X_{ij}\right)$ can be obtained by equation (3).


(3) $$v_{i}^{T}\bar{v_{j}}+b_{i}+\bar{b_{j}}=\log\left(X_{ij}\right)$$

The loss function of the Glove model is shown in equation (4).


(4) $$J=\overset{V}{\underset{i=1}{\sum }}\overset{V}{\underset{j=1}{\sum }}f\left(X_{ij}\right){\left(v_{i}^{T}v_{j}+b_{i}+b_{j}-\log\left(X_{ij}\right)\right)}^{2}$$

f(x)is shown in equation (5).


(5) $$f\left(x\right)={\{\begin{array}{c} \left(\frac{x}{x_{\max}}\right)\\ 1,othrewise \end{array}}^{a}$$

In equations (4–5), Vrepresents the size of the task corpus, $v_{i}$ is the current word vector, $v_{j}$ is the word vector appearing in the window, $b_{i},b_{j}$ is the offset value, a and $x_{\max}$are parameters set according to the task requirements, and ${\left(v_{i}^{T}v_{j}-\log\left(X_{ij}\right)\right)}^{2}$ is the mean square error.The Glove model uses the ratio of probabilities to represent the correlation between words and uses only the co-occurrence matrix of The Glove model uses the ratio of probabilities to represent the correlation between words and uses only non-zero elements in the co-occurrence matrix as samples for training, which can effectively use the statistical information of words, and in the experiments of the authors of the paper, the Glove model works better than Word2vec (Wang, 2017).

### Deep reinforcement learning

Deep Reinforcement Learning (DRL) is formed by the combination of deep neural network with strong perception ability and traditional reinforcement learning method with strong decision-making ability, among which the most famous deep neural network includes Convolutional Neural Network (CNN), Long Short-Term Memory Networks (LSTM), Recurrent Neural Networks (RNN), and Autoencoders. Deep reinforcement learning first uses the deep learning network as a function approximator (FA) to fit the parameters required for reinforcement learning, and then uses reinforcement learning to realize decision-making, in which the deep neural network is used to represent the value function (Q-Learning), Policy Optimization or Environment Model (Figure 3).

**Figure 3:** Deep reinforcement learning process.

When people observe something, they naturally focus their attention on a certain area in their visual field, which usually has more important information than other areas. This approach helps people to quickly find what they are interested in from the large amount of information in the limited visual field and improves the efficiency of the brain in processing information.

### Circulatory neural network and its variants

The original neural network stipulates that the neurons in the input layer are independent of each other and do not communicate with each other, and each layer is connected only by weighting, but in fact the input of text is semantically related to each other. RNN is derived from this. In order to clearly show the concrete structure of the model, this paper expands the model structure. The expanded model structure mainly includes input layer, hidden layer and output layer. The calculation process of the result $y_{t}$ obtained by the output layer at the final moment t is shown in equation (6), in which softmax is used to normalize the result.


(6) $$y_{t}=soft\max\left(Vs_{t}\right)$$

Although RNN is a classic chain structure, in practice, gradient disappearance and gradient explosion often occur after backpropagation. In order to alleviate this situation, scholars try to make certain improvements on the basis of RNN., resulting in many models (Han et al., 2016; Zhu, 2017; Hou et al., 2019). It can be seen that the hidden unit of the RNN is appropriately changed, and a gating mechanism is added. This gating mechanism is called a memory cell. The model controls and judges whether the information is useful and realizes the information through the gating mechanism. Additions, updates and deletions.

### Activation functions

Many real-life tasks cannot be fully processed by linearization. For neural network models, an activation function is often used to transform the output of the neural network in a nonlinear way, which gives the neural network the ability to capture nonlinear information in the data. This approach makes the neural network more capable of fitting the actual task and also enhances the learning ability of the neural network. The more common activation functions at present are Sigmoid, tanh, and Relu.

Sigmoid maps the output value into the (0,1) interval by nonlinear means. This model is a maximum entropy model, which is less affected by noisy data, and the model is easy to handle, and its derivatives can be obtained relatively easily. However, the model in the use of the gradient saturation phenomenon, when the value is too large or too small gradient will be close to 0, which will lead to slow training progress or even cause the gradient disappearance of the occurrence. At present, this function is widely used in dichotomous classification-related tasks.

The formula of Sigmoid is shown in equation (6).


(7) $$Sigmoid\left(x\right)=\frac{1}{1+e^{-x}}$$

Although tanh function can improve the convergence speed of neural network, it still cannot avoid the problem of gradient disappearance in the training process of neural network. However, tanh function solves the problem that Sigmoid is not zero-centered, and it will achieve better results in tasks with obvious differences in features. The formula of tanh is shown in equation (8).


(8) $$\tanh=\frac{1-e^{-2x}}{1+e^{2x}}$$

When the value of Relu is positive, the gradient value will always be 1, which effectively solves the problem of gradient disappearance in Sigmoid, tanh and other models. The formula of Relu is shown in equation (9), and the effect of Relu is shown in Figure 4.

**Figure 4:** Schematic diagram of Relu.

However, Relu also has certain drawbacks. When the output value of the neural network is distributed in the negative range, the gradient value will always remain at the 0 value, which will cause the problem that the weight cannot be updated continuously. In order to effectively alleviate this problem, PReLU (ParametricRectifiedLinearUnit), which adds a new parameter a on the basis of Relu, where a < 0, this parameter can be continuously adjusted with the training process, the formula of PReLU is such as equation (9) As shown, in the current practical application process, Relu and PReLU are widely used.


(9) $$\sigma =\{{}_{x,x>0}^{ax,x<0}$$

It is used to deal with overfitting problems that often occur in neural network models. The core idea of this technology is that a certain number of neurons in the hidden layer will be disconnected in every training process of neural network, and this operation is completely random. The output of neurons in the hidden layer to be discarded in the model is set to 0, and the weights of these selected neurons will stop updating in this training process. It is worth noting that all neurons will participate in the work in the final testing process. Dropout can reduce the degree of interaction between hidden layer nodes, and keep certain generalization ability in different features.

## Empirical study design

### Sentiment analysis model based on custom classifier

The problem of how to integrate user and product information into sentiment analysis is also a question worth considering.

This chapter combines the DBi LSTM with the DBi LSTM. In this chapter, we combine DBi LSTM and self-attention network layers to capture deep text features and semantic relationships. The input temporal data is trained by DBi LSTM, and the final layer output values are further extracted by self-attention to extract important features and semantic relationships. Considering the influence of user information and product information on the analysis results, the model combines user information and product information to build a custom classifier, which formulates specific parameters for user information and product information through context-aware attention, and processes and analyzes the extracted text features together with the original parameters. The experimental results on three common datasets in this chapter can show that the feature extraction scheme of DBi LSTM model combined with self-attention mechanism proposed in this chapter can effectively extract text features, and the classifier constructed in this chapter can improve the analysis accuracy.

#### CNN

A classical convolutional neural network, which performs classification tasks through convolution calculation and pooling.

#### AT-Dou CNN

Use attention mechanism to enrich the feature information of word vectors, then extract features through multiple convolution kernels, use maximum pool to screen out the most prominent features, then use full connection layer to merge the features of two channels, and finally use softmax function to output the classification results.

Figure 5 depicts the variation curve of the accuracy rate during the training of the three ATT-based models during the experiment. The three models use the same learning rate. It can be seen from the figure that the convergence speed of the ATT-C-LSTM model is slightly slower than that of AT-DouCNN. To solve the problem of insufficient ability of extracting text feature information by using convolutional neural network and cyclic neural network, a Capsule-Attention emotion analysis model is proposed. In this model, word2vec technology is used to process text information into word vectors, feature extraction of word vectors is carried out by using capsule network, and then self-attention mechanism is introduced to weight key words, and the final classification result is obtained. Several sets of benchmark models are set up, and the comparative experiment and ablation experiment are carried out. The experimental results show that this model can achieve good classification effect when it comes to emotion classification, and it shows excellent performance compared with other mainstream emotion analysis models.

**Figure 5:** Accuracy results of the model during training period graph.

### Hierarchical network sentiment analysis model based on attentional interaction mechanism

In this chapter, the number of cells per layer of DBi LSTM is set to 256, the number of word vectors is set to 300, and the number of user vectors and product vectors is set to 64. To prevent overfitting, dropout and early stopping regularization methods are used in the training process. To prevent gradient explosion, gradient clipping is used to control the training process. In order to verify the effectiveness of the model, the accuracy and the mean square error (RMSE) are used as the model measures in the experiments. Accuracy is an assessment of the model’s ability to analyze correctly, and the higher the accuracy, the better the result. rMSE is a measure of the difference between the true and predicted values, and the smaller the value of this indicator, the better the result (Figures 6, 7).

**Figure 6:** RMSE value graph.

**Figure 7:** Accuracy diagram.

The dynamic routing idea is the most essential difference between the capsule network and other neural networks. In the capsule network, the clustering transfer of features is accomplished between the lower-level capsule and the higher-level capsule by a dynamic routing algorithm, and the number of routes of the dynamic routing algorithm is directly related to the model’s ability to extract features, and the different number of routes affects the classification effect of the model. Therefore, it is necessary to set up a control experiment in order to determine the optimal number of routes. According to the figure, during the training process, as the number of iterations of inter-capsule layer routing increases, the accuracy of the model classification rises first and then falls, and the loss falls first and then rises, and the model performs best when the number of iterations is 5.0. When the number of iterations is too small, no effective routing relationship can be established between the layers of capsules, and the prediction vector of the lower layer capsules corresponding to the presumed higher layer capsules is too short in its mode length due to the lack of feature information to accurately represent the features. Since the higher-level capsule is a weighted sum among the lower-level capsules, as the number of iterations increases, the features learned in the capsule layer may not play a proper role due to their too short modal lengths due to clustering, and the generalization of the model decreases, leading to performance degradation. Through the analysis of the results of the above ablation experiments, it can be verified that each strategy in the model proposed in this chapter contributes to the final classification effect, and it is also verified that the overall model performance can be further improved when multiple strategies are combined.

### MCNN-Cap Net-LSTM model based on multiple convolution kernels

Capsule network (Caps Net) can generalize the same object from different perspectives in different 3D images. It is mainly used in the direction of computer vision and less in the direction of natural language processing. This chapter details the structure of the capsule network. Modification, on this basis, a MCNN-Cap Net-LSTM model is proposed. The model first uses the characteristics of the convolutional neural network (CNN) to extract the n-gram features of words through multiple convolution kernels, and then merge and extract them into The n-gram features of the network are clustered through the capsule network, and then the context information of important features is extracted through the long short-term memory network (STM), the unimportant information is discarded, and the sentiment analysis is completed. Experiments show that MCNN-Caps Net-LSTM It has better performance than other models in sentiment classification tasks (Figure 8).

**Figure 8:** Experimental results of loss rate of model classification under different routing times.

Ext CNN applies convolutional network to sentiment classification, which uses convolution to learn n-gram features of word vectors, and then splices the most prominent features by maximum pooling of the convolutionally extracted feature maps, which has good results in sentiment analysis tasks (Yang, 2020). The MCNN-Caps Net-LSTM model is based on the idea of dynamic routing and uses coupling coefficients to weight the average of all the extracted features, taking into account the role of each feature, unlike maximum pooling, which only retains one feature. The disadvantage of losing feature information in pooling pools is overcome to a certain extent. Therefore, MCNN-Caps Net-LSTM is more effective than Text CNN.

Although the BGCapsule, BGRU + Capsules, and Caps Net-GRU-Attention models use the gating mechanism to replace the pooling layer in the convolutional neural network, and its superiority over the Text CNN model has been experimentally verified to overcome the disadvantages of the convolutional neural network to a certain extent, the MCNN-Caps Net-LSTM model The dynamic routing idea used can also avoid the problem of feature loss in the convolutional layer, and the MCNN-Caps Net-LSTM model can also extract the contextual information, so the MCNN-Caps Net-LSTM model performs better than them on the sentiment analysis task. The results of the study show that the accuracy of the algorithm in this paper is high, and its reduction is about 5% compared with the traditional algorithm. The method can reduce the number of iterations and the running time of the algorithm.

## Conclusion

Traditional methods for sentiment analysis are sentiment knowledge base based methods and machine learning based methods. In recent years, deep learning has been the focus of research in the field of artificial intelligence, and many studies have shown that deep learning has better performance than traditional methods in the field of NLP. In this paper, we collect and summarize the existing research done in the field of sentiment analysis at home and abroad, mainly focusing on the psychological feature analysis and emotional expression of deep learning in higher education music education using deep learning methods to try to build a sentiment analysis algorithm model to improve the analysis effect of text sentiment analysis, with the development of deep learning in recent years, many neural network-based models have achieved good results, but there are still some One is that neural networks learn feature information through word vectors, while existing methods seriously underutilize the feature information of Chinese words and cannot focus on key words. Second, many convolutional neural network-based models still have the defect of losing feature information. The attention mechanism gives more attention to the focus region in the model, and applying the attention mechanism to the sentiment classification problem can enable the model to focus on the focus words and learn the complex semantic relationships. This paper firstly describes the research background and research significance of recommendation system, and analyzes and compares the research status of domestic and foreign research. With the rapid development of online education, the research of recommendation algorithms is also new, but most of them are based on traditional recommendation algorithms and are not applied to various platforms on a large scale, and information overload is still an important problem in online education. In this paper, we propose a deep learning based psychological feature analysis and emotion expression algorithm in higher education music education, and use it as the core to design and implement a deep learning based psychological feature analysis and emotion expression system in higher education music education, by using this system, we can solve problems for students. The research results show that the accuracy of the algorithm in this paper is high, and its reduction is about 5% compared with the traditional algorithm. The method can reduce the number of iterations and the running time of the algorithm.

## Data availability statement

The original contributions presented in the study are included in the article/supplementary material, further inquiries can be directed to the corresponding author.

## Author contributions

The author confirms being the sole contributor of this work and has approved it for publication.

## Conflict of interest

The author declares that the research was conducted in the absence of any commercial or financial relationships that could be construed as a potential conflict of interest.

## Publisher’s note

All claims expressed in this article are solely those of the authors and do not necessarily represent those of their affiliated organizations, or those of the publisher, the editors and the reviewers. Any product that may be evaluated in this article, or claim that may be made by its manufacturer, is not guaranteed or endorsed by the publisher.
